RETRACTED

# Study on the Mechanism of miR-34a Affecting the Proliferation, Migration, and Invasion of Human Keloid Fibroblasts by Regulating the Expression of SATB1

**DOI:** 10.1155/2021/8741512

**Published:** 2021-09-28

**Authors:** Lei Jiang, Xiufang Shi, Meng Wang, Huaxia Chen

**Affiliations:** ^1^Shandong University, Jinan, China; ^2^Department of Burn and Plastic Surgery, Yantai Yuhuangding Hospital Affiliated to Qingdao University, Yantai, Shandong 264000, China; ^3^Operation Room of West Zone, Yantai Yuhuangding Hospital Affiliated to Qingdao University, Yantai, Shandong 264000, China

## Abstract

**Objectives:**

To explore the effect and mechanism of miR-34a on the proliferation, migration, and invasion of keloid fibroblasts (KFB).

**Methods:**

Isolate and culture KFB and normal skin fibroblast (NFB), detect the mRNA expression levels of miR-34a and integrin *β*5 (SATB1) in KFB and NFB by RT-qPCR, and detect SATB1 by western blot. The level of protein expression, MTT method, Transwell method, RT-qPCR, and western blot were used to detect the effects of overexpression of miR-34a or inhibition of SATB1 expression on the proliferation, migration, and invasion of KFB cells and the expression of related proteins. The dual luciferase reporter gene test verifies the targeting relationship between miR-34a and SATB1.

**Results:**

Compared with NFB, the expression of miR-34a was downregulated in KFB and the mRNA and protein expression levels of SATB1 were upregulated. Overexpression of miR-34a or inhibition of SATB1 expression inhibited the proliferation, migration, and invasion of KFB. miR-34a can negatively regulate the expression of SATB1, and overexpression of SATB1 reverses the effects of overexpression of miR-34a on the proliferation, migration, and invasion of KFB.

**Conclusions:**

miR-34a inhibits the proliferation, migration, and invasion of keloid fibroblasts by downregulating the expression of SATB1.

## 1. Background

Keloid is a skin fibrotic disease characterized by excessive proliferation of fibroblasts and excessive precipitation of extracellular matrix such as collagen [1]. The pathogenesis of keloids is not yet clear, and there is a lack of satisfactory therapeutic drugs [2]. The treatment of keloid scars is mainly surgical resection, but the treatment effect is poor and it is easy to relapse [3]. Therefore, it is of great significance to explore the pathogenesis of keloids and find a target for effective treatment of keloids. MicroRNA (miRNA) is a type of small noncoding RNA with a length of 21–25 nucleotides. It can bind to specific mRNA or regulate gene expression by regulating the protein translation process of specific mRNA [4].

RETRACTED

In recent years, some scholars have studied miRNA expression profiles in keloids and normal skin and found multiple differentially expressed miRNAs. The upregulated miRNAs include miR-1202, miR-1207, miR-21, miR-130, and miR-1915, and the downregulated ones include miR-451 and miR-720. Bioinformatics further analyzed that these differentially expressed miRNAs are related to many important factors in the process of scar formation, including collagen formation, fibroblast growth factor, transforming growth factor, platelet-derived growth factor, and insulin-like growth factor. Studies have found that miR-200b is significantly downregulated in hypertrophic scar tissue and scar skin fibroblasts, and miR-200b can affect the proliferation and apoptosis of scar skin fibroblasts and regulate the expression of collagen genes I and III. This study intends to study the specific mechanisms of miR-34a and SATB1 mediating the proliferation, migration, and invasion of keloid fibroblasts.

## 2. Materials and Methods

### 2.1. Materials

Fetal bovine serum (FBS) and DMEM medium were purchased from Gibco, US; MTT was purchased from Amresco, US; Lipofectamine TM 2000 kit was purchased from Invitrogen, US; miR-34a mimic (mimic), mimic negative control, miR-34a inhibitor (anti-miR-34a), negative control sequence (anti-miRNA-NC), SATB1 small interfering RNA (si-SATB1), and scrambled nonsense negative sequence (si-NC) were purchased from Guangzhou Ruibo Biotech Company; Trizol reagents and reverse transcription kits were purchased from Fermentas, USA; PCR kits were purchased from Dalian Bao Biological Co., Ltd.; and primer sequences were designed and synthesized by Shanghai Bioengineering Company.

### 2.2. Cultivation of KFB and Normal Skin Fibroblast (NFB)

Take fresh keloids and healthy human normal skin tissue specimens, which are soaked in 0.5% chlorhexidine solution for 5 min, rinsed with normal saline 3 times, and then cut into pieces, placed in a Petri dish, and added with 20% FBS. The DMEM medium is placed in an incubator at 37°C, 5% CO_2_, and 97% humidity. Change the culture medium every 2 to 3 days, and observe using the phase contrast microscope. When the cells swim out and the fusion takes up about 80% of the bottom area of the Petri dish, they are passaged. Subsequent experiments use 4 to 7 passages of cells.

### 2.3. Cell Transfection

Take the KFB in the logarithmic growth phase, and inoculate it in a 6-well plate. When the cells grow to 60%, refer to the Lipofectamine TM 2000 kit instructions to separately compare miR-34a mimic (miR-34a group) and mimic negative control (miRNA-NC group); miR-34a mimics and pcDNA (miR-34a + pcDNA group); and miR-34a mimics and pcDNA-SATB1 (miR-34a + pcDNA-SATB1 group) transfected into KFB. At the same time, a blank control group was set, KFB did not perform any operation, and cultured normally. Cells were collected 48 h after transfection for subsequent experiments.

RETRACTED

### 2.4. MTT Detects Cell Proliferation

Each group of KFB was made into a single cell suspension, inoculated in a 96-well plate at 2.5 × 10^4^ cells/ml, 200 *μ*l per well, and cultured for 24, 48, and 72 h, and 3 replicate wells were set for each group. After the incubation, add 20 *μ*l of 5 mg/ml MTT solution to each well and continue to incubate for 4 h. Discard the supernatant, add 150 *μ*l dimethyl sulfoxide to each well, react for 10 min, mix well, and measure the absorbance (A 490) at 490 nm with a microplate reader. The experiment was repeated three times.

### 2.5. Transwell Detects Cell Migration Ability

KFB of each group was inoculated into the upper chamber of Transwell cell at 1 × 10^5^ pieces/ml, 100 *μ*l per well. There are 3 replicate holes in each group. Add 500 *μ*l of DMEM medium containing 10% FBS to the lower chamber. After culturing for 48 hours, the culture medium was aspirated and the upper chamber was taken out, fixed with 4% paraformaldehyde, stained with crystal violet, and observed with an inverted microscope. Randomly select 5 fields of view to calculate the number of migrating cells. The cell migration ability is expressed by the number of cells passing through the filter membrane into the lower chamber. The experiment was repeated three times.

### 2.6. Transwell Detects Cell Invasion Ability

The upper chamber of the Transwell chamber is covered with Matrigel glue as an invasion model, and the rest of the operation is the same as the cell migration test. The number of cells passing through the filter membrane into the lower chamber represents the invasion ability of the cells.

### 2.7. RT-qPCR Detects the mRNA Expression Levels of miR-34a and SATB1

Each group of KFB was seeded in a 24-well plate at 2.5 × 10^4^ cells/ml per well. After 48 hours of culture, trypsin digestion was performed to collect the cells of each group. Trizol reagent lyses cells to extract total RNA, and reverse transcription of RNA into cDNA was performed using a reverse transcription kit. Using cDNA as a template, refer to the operating instructions of the PCR kit for amplification. The PCR amplification conditions are as follows: 95°C predenaturation for 30 s, 95°C denaturation for 5 s, 60°C annealing for 30 s, and 72°C extension for 30 s, a total of 45 cycles. miR-34a uses U6 as the internal control, SATB1 uses GAPDH as the internal control, and the relative expression levels of miR-34a and SATB1 mRNA are calculated by the 2^−△△Ct^ method.

RETRACTED

### 2.8. Western Blot Detection of Protein Expression

Detect the expression of related proteins in the cell. Each group of KFB was inoculated into a 24-well plate at 2.5 × 10^4^ pieces/ml per well. After 48 hours of culture, the cells were trypsinized, and the cells of each group were collected. The lysis buffer was added and placed on ice for full lysis. Centrifuge at 10000 r/min for 10 min, take the supernatant, and determine the protein concentration by the BCA method. After SDS-PAGE electrophoresis, the total protein was transferred to a polyvinylidene fluoride membrane and blocked with 5% skim milk at room temperature for 2 hours. After washing the membrane with TBST, add the primary antibody and incubate overnight at 4°C in the refrigerator. Wash the membrane with TBST, add the secondary antibody, and continue to incubate at 37°C for 1 h. After washing the membrane with TBST, add ECL to develop, expose, and take pictures. Image J1.8.0 software measures the gray value of the internal reference protein GAPDH and the protein band to be tested. The expression of the test protein is expressed by the ratio of the gray value of the test protein to the internal reference protein. Verification of the targeting relationship between miR-34a and SATB1: bioinformatics software predicts that there are binding sites between the 3′UTR of SATB1 and the nucleotide sequence of miR-34a. The 3′UTR sequence of SATB1 containing miR-34a binding site was amplified by PCR to construct SATB1 wild-type (WT-SATB1) and mutant (MUT-IT-GB5) luciferase reporter plasmids. WT-SATB1, MUT-SATB1, and miR-34a mimics or miRNA-NC were transfected into KFB, respectively. After 48 h of transfection, refer to the luciferase detection kit operating instructions and bioluminescence instrument to detect luciferase activity. Simultaneously transfect miR-34a mimics (miR-34a group) and miRNA-NC (miRNA-NC group). After transfection into KFB 48 hours, trypsin digestion, harvest the cells and western blot to detect the expression level of SATB1 protein in the cells.

### 2.9. Statistical Methods

The experimental data use SPSS22.0 software for statistical analysis. The measurement data are expressed by mean ± SD, the independent sample *t* test is used for the comparison between the two groups, and the single-factor analysis of variance is used for the comparison between multiple groups. *P* < 0.05 indicates that the difference is statistically significant.

## 3. Results

### 3.1. The Expression of miR-34a and SATB1 in KFB and NFB

Compared with NFB, the expression level of miR-34a in KFB was significantly reduced (*P* < 0.05), and the expression levels of SATB1 mRNA and protein were significantly increased (*P* < 0.05), indicating that the expression of miR-34a in KFB was downregulated and that of SATB1 was upregulated. Note the expression of miR-34a in KFB and NFB, the expression of SATB1 mRNA in KFB and NFB, and the expression of SATB1 protein in KFB and NFB in Figure 1.

RETRACTED

### 3.2. The Effect of miR-34a Overexpression on the Proliferation of KFB

The level of miR-34a in KFB in the miR-34a group was significantly higher than that in the miRNA-NC group (*P* < 0.05), indicating that miR-34a mimics were successfully transfected and miR-34a was overexpressed in KFB. Compared with the miRNA-NC group, the A 490 value of KFB in the miR-34a group was significantly reduced after 48 h and 72 h of culture (*P* < 0.05), cyclinD1 protein level was reduced (*P* < 0.05), and *p*21 and *p*27 protein level increased (*P* < 0.05). There was no significant difference between the blank control group and the miRNA-NC group in the detection indicators (*P* > 0.05). See Figure 2 for details.

### 3.3. The Effect of miR-34a Overexpression on KFB Migration and Invasion

Compared with the miRNA-NC group, the number of KFB migration and invasion in the miR-34a group was reduced (*P* < 0.05), and the protein expression of MMP-2, MMP-9, and MMP-14 was significantly reduced (*P* < 0.05). There was no significant difference between the blank control group and the miRNA-NC group in the detection indicators (*P* > 0.05); see Figure 3 for details.

### 3.4. miR-34a Targets and Regulates the Expression of SATB1

Compared with the miRNA-NC group, the KFB luciferase activity of the miR-34a group carrying the WT-SATB1 reporter gene carrier was significantly reduced (*P* < 0.05), while the KFB luciferase carrying the MUT-SATB1 reporter gene carrier, there was no significant change in activity (*P* > 0.05). The protein level of SATB1 in the miR-34a group was significantly lower than that in the miRNA-NC group (*P* < 0.05). See Figure 4 for details.

## 4. Discussion

Keloid is a common skin fibrous tissue hyperplasia disease, which is mainly related to the abnormal proliferation of fibroblasts and abnormal collagen synthesis [5–7]. There are many treatment methods for keloid scars, but the effect is poor. With the rapid development of genetic engineering, fibroblasts are induced in a targeted manner through genetic engineering methods.

miRNA mainly acts as a tumor suppressor or oncogene by acting on target genes. Bioinformatics studies have found that the 3′UTR of SATB1 contains a nucleotide sequence complementary to miR-34, suggesting that miR-34 may target and regulate SATB1 expression. Previous studies have proved that SATB1 can interact with some transcription factors and chromatin histone modifying enzymes and can bind to special DNA sequences, regulate gene expression, and participate in the regulation of various physiological functions of the organism. As a highly conserved miRNA, miR-34a is also involved in the regulation of a variety of biological events in cells: (1) cell cycle arrest [8]. (2) Promote cell senescence [9]: the introduction of miR-34a and miR-34b/c into human fibroblasts will cause cell aging. A study transfected miR-34a into HCT116 cells, RKO cells, and *p*53 mutant SW480 cells and found that the cell size increased and caused senescence and related galactosidase (senescence-associated galactosidase) was positive, indicating that miR-34a can induce cell senescence. (3) Induce cell apoptosis [10]: miR-34s reactivates in cancer cells, promotes the cleavage of caspase3 and PARP, and induces caspase-regulated apoptotic pathways. (4) Prevent cell migration [11]: in melanoma and liver cancer tissues, the reactivation of miR-34 can inhibit c-Met protein and prevent tumor cell migration and infiltration [11].

RETRACTED

The results of the luciferase reporter gene test in this study showed that miR-34a mimic can reduce the luciferase activity of SATB1 wild-type, but has no significant effect on the mutant luciferase activity, suggesting that miR-34 can be compared with the 3′ UTR of SATB1 targeted binding sites. In addition, after upregulating the expression of miR-34 in KFB, the expression of SATB1 protein was downregulated, and after downregulating the expression of miR-34, the expression of SATB1 protein was upregulated, further confirming that miR-34 in KFB can negatively regulate the expression of SATB1. This study also showed that overexpression of SATB1 reversed the effects of overexpression of miR-34 on the proliferation, migration, and invasion of KFB, suggesting that overexpression of miR-34 inhibits the proliferation, migration, and invasion of KFB by targeting the expression of SATB1. One miRNA can often simultaneously regulate multiple target genes with the same target site.

The level of miR-34a in KFB in the miR-34a group was significantly higher than that in the miRNA-NC group (*P* < 0.05), indicating that miR-34a mimics were successfully transfected and miR-34a was overexpressed in KFB. Compared with the miRNA-NC group, the A 490 value of KFB in the miR-34a group was significantly reduced after 48 h and 72 h of culture (*P* < 0.05), cyclinD1 protein level was reduced (*P* < 0.05), and *p*21 and *p*27 protein level increased (*P* < 0.05). There was no significant difference between the blank control group and the miRNA-NC group in the detection indicators (*P* > 0.05). Compared with the miRNA-NC group, the number of KFB migration and invasion in the miR-34a group was reduced (*P* < 0.05), and the protein expression of MMP-2, MMP-9, and MMP-14 was significantly reduced (*P* < 0.05). There was no significant difference between the blank control group and the miRNA-NC group in the detection indicators (*P* > 0.05). Compared with the miRNA-NC group, the KFB luciferase activity of the miR-34a group carrying the WT-SATB1 reporter gene carrier was significantly reduced (*P* < 0.05), while the KFB luciferase carrying the MUT-SATB1 reporter gene carrier, there was no significant change in activity (*P* > 0.05). The protein level of SATB1 in the miR-34a group was significantly lower than that in the miRNA-NC group (*P* < 0.05). Compared with NFB, the expression level of miR-34a in KFB was significantly reduced (*P* < 0.05), and the expression levels of SATB1 mRNA and protein were significantly increased (*P* < 0.05), indicating that the expression of miR-34a in KFB was downregulated and that of SATB1 was upregulated.

RETRACTED

In summary, miR-34 is underexpressed in KFB and overexpression of miR-34 can inhibit the proliferation, migration, and invasion of KFB. SATB1 is the target gene of miR-34, and miRNA-143-3p may play a role by downregulating the expression of SATB1.

## Figures and Tables

**Figure 1:** Expression of miR-34a and SATB1 in KFB and NFB. (a) mRNA expression levels of miR-34a and SATB1 in NFB and KFB, respectively; (b) protein expression levels of SATB1 in NFB and KFB, respectively. ^*∗*^*P* < 0.05.

**Figure 2:** The effect of miR-34a overexpression on the proliferation of KFB and related proteins. (a) mRNA expression after miR-34a overexpression; (b) cell viability after miR-34a overexpression; and (c) cyclinD1, *p*21, and *P*27 protein expression after miR-34a overexpression. ^*∗*^*P* < 0.05.

**Figure 3:** The effect of miR-34a overexpression on KFB migration and invasion and related proteins. (a) Cell migration and invasion after miR-34a overexpression and (b) comparison of protein expression levels of MMP-2, MMP-9, and MMP-14 after miR-34a overexpression. ^*∗*^*P* < 0.05.

**Figure 4:** miR-34a targets the expression of SATB1. (a) Bioinformatics analysis shows that SATB1 and miR-34a are mutual interaction targets and (b) luciferase activity detection result after SATB1 mutation. ^*∗*^*P* < 0.05.

## Data Availability

The original data could be obtained from the corresponding author.
